The article "Cerium oxide nanoparticle-loaded polyvinyl alcohol nanogels delivery for wound healing care systems on surgery" was retracted in 2023. Reasons: lack of ethics approval or compliance; concerns about the data; concerns about the results or conclusions.

# Cerium oxide nanoparticle-loaded polyvinyl alcohol nanogels delivery for wound healing care systems on surgery

**DOI:** 10.1080/10717544.2020.1858998

**Published:** 2021-02-17

**Authors:** Lianlian Cao, Guojing Shao, Fengmei Ren, Minghua Yang, Yan Nie, Qian Peng, Peng Zhang

**Affiliations:** a Emergency Department, Dongying People’s Hospital, Dongying, China; b Psychiatry Department, Dongying Rongjun Hospital, Dongying, China; c Health Care Department, Dongying People’s Hospital, Dongying, China

**Keywords:** Cerium nanogels, polyvinyl alcohol, wound healing, *in vivo* mouse model

## Abstract

This study was designed to establish the composition of wound bandages based on Cerium nanoparticle (CeNP)-loaded polyvinyl alcohol (PVA) nanogels. The CeNP nanogel (Ce-nGel) was fabricated by the fructose-mediated reduction of Cerium oxide solutions within the PVA matrix. The influences of different experimental limitations on PVA nanogel formations were examined. The nanogel particle sizes were evaluated by transmission electron microscopy and determined to range from ∼10 to 50 nm. Additionally, glycerol was added to the Ce-nGels, and the resulting compositions (Ce-nGel-Glu) were coated on cotton fabrics to generate the wound bandaging composite. The cumulative drug release profile of the Cerium from the bandage was found to be ∼38% of the total loading after two days. Additionally, antibacterial efficacy was developed for Gam positive and negative microorganisms. Moreover, we examined *in vivo* healing of skin wounds formed in mouse models over 24 days. In contrast to the untreated wounds, rapid healing was perceived in the Ce-nGel-Glu-treated wound with less damage. These findings indicate that Ce-nGel-Glu-based bandaging materials could be a potential candidate for wound healing applications in the future.

## 1. Introduction

Wound dressings serve as adjuncts to the wound healing process by providing favorable conditions at the site of injury. An ideal wound dressing would be one with excellent antimicrobial nature, tissue compatibility, gas permeability, effective exudate absorption and accelerated healing process (Yu et al., 2016; Bakshi, 2017; Memic et al., 2019). Therefore, it is highly desirable to design a high-performance antibacterial wound care system that would effectively enhance the wound healing process. Hydrogels have shown enormous potential in the development of wound care systems due to their high exudate absorptive capacity and biocompatibility. It has been shown that wound healing is faster under a wet environment due to the greater mobility of the extracellular matrix components (Liu et al., 2018; Nethi et al., 2019; Son et al., 2019). Additionally, hydrogels may be peeled off without any damage to the regenerated surface obviating trauma to the patient (Shen et al., 2020; Zhao et al., 2020a).

The article "Cerium oxide nanoparticle-loaded polyvinyl alcohol nanogels delivery for wound healing care systems on surgery" was retracted in 2023. Reasons: lack of ethics approval or compliance; concerns about the data; concerns about the results or conclusions.

Enormous studies have been carried out to develop wound dressings based on a large number of polymers. Dressings based on PVA hydrogel are widely favored for wound management due to composite features of biocompatibility and hydrogel nature (Qu et al., 2018; Liang et al., 2019, 2020; Zhao et al., 2020b). Agarwal et al. developed drug-loaded PVA-carboxymethyl cellulose-polyethylene oxide membranes for efficient wound management. The efficiency of ciprofloxacin, aloe vera, and curcumin loaded wound dressings toward wound healing was investigated. PVA-polysaccharide gels have been proposed by crosslinking using gamma radiation. (Sekhon & Sen Gupta, 2018; Deal et al., 2020; Sener et al., 2020; Thapa et al., 2020). Clinical trials showed that such gels can be effectively used to treat burn wounds, healing impaired ulcers, leprosy and other external wounds. Organically modified montmorillonite clay incorporated PVA wound dressings have also been developed and were found to show excellent physical and mechanical properties. On the other hand, PVA/povidone electrospun nanofibrous mats have been investigated for wound healing applications (Hamdan et al., 2017; Ma et al., 2020; Thongsuksaengcharoen et al., 2020). Flexible dressings were obtained by using a combination of chitosan/polyvinyl pyrrolidone/polyethylene glycol on the cotton fabric. Nonwoven viscose fabrics coated with chitosan and PVA have also exhibited complete wound healing and reepithelialization during *in vivo* studies (Hu & Xu, 2020).

Incorporation of an antimicrobial agent is necessary to prevent infection at the wound site and to enhance the wound healing efficiency of hydrogel systems. Although a wide variety of antimicrobial agents are available, antibiotic resistance of microorganisms poses a major problem, resulting in complications such as delayed wound healing. In recent years, extensive research has been dedicated to the development of nanosilver based systems due to its high effectiveness against microbes. Anisha et al. reported the development of chitosan–hyaluronic acid/nanosilver composite sponge-based wound dressing for diabetic foot ulcers infected with drug-resistant bacteria. Chitin/nanosilver based scaffolds with exceptional antimicrobial activity have been fabricated for potential use in wound management. Furthermore, hydrogel systems based on polyvinyl pyrrolidone/alginate containing Cerium with efficient fluid handling capacity and antimicrobial activity have been developed for wound dressing applications (Hartwell et al., 2011; Tu et al., 2019; Xu et al., 2019; Gao et al., 2020). Chitin-covered CeNPs have also demonstrated promising wound management. Additionally, the hydrogels based on alginate-coated PVA and polyvinyl pyrrolidone with CeNPs have shown promising fluid absorption capabilities and antimicrobial properties (Sakai et al., 2013; Song et al., 2016; Wang et al., 2016; Thakar et al., 2019; Deng et al., 2020).

The article "Cerium oxide nanoparticle-loaded polyvinyl alcohol nanogels delivery for wound healing care systems on surgery" was retracted in 2023. Reasons: lack of ethics approval or compliance; concerns about the data; concerns about the results or conclusions.

In the present work, we attempted to develop PVA and CeNPs based wound dressings. The study was formulated with a 2-fold objective. In the first step, synthesis and characterization of the CeNPs within the PVA matrix (Ce-nGel) was carried out using fructose as the reducing agent. Glycerol, a biocompatible material, was introduced in the Ce-nGel composition to develop Ce-nGel-Glu composition. The Ce-nGel and Ce-nGel-Glu were coated on cotton fabric to develop composite matrices. Subsequently, the wound healing efficacies of Ce-nGel and Ce-nGel-Glu treated cotton fabrics were evaluated using *in vitro* antimicrobial testing and *in vivo* animal testing.

## 2. Experimental section

### 2.1. Materials

Cerium oxide solutions, β-D-Fructose (J&D, China), glycerol (J&D, China), and PVA (Mw ∼ 1,50,000, S D Fine Chemicals, India) were used in the synthesis of nanogels. Luria broth and agar-agar, were obtained from Hi Media Laboratories, India. Bacterial strains of E. coli and S. aureus were provided by institutions. All chemicals were of analytical grade and used without further purification. Cotton fabric (21.24 GSM and 67% porosity) was separated from Surgipad dressings manufactured by Johnson & Johnson Limited. Ultra-pure water (18 MΩcm) from Millipore Milli-Q system was used in all experiments.

### 2.2. Fabrication of Ce-nGel and Ce-nGel-Glu

To 50 mL 0.1% PVA solution containing 0.01 g of fructose, 50 mL of 100 ppm Cerium oxide solution was added dropwise under continuous stirring for predetermined time intervals at temperatures in the range of 60–90 °C. The weight ratio of AgNO3 to fructose was maintained 1:1. Ce-nGel-Glu was prepared by mixing nGel with 20% (v/v) glycerol.

### 2.3. Characterization of Ce-nGel and Ce-nGel-Glu

The formation of CeNPs in the colloidal solution was monitored using a Perkin Elmer Lambda 35 UV-Vis spectrophotometer at wavelengths between 200 and 600 nm. The free Cerium band at ∼300 nm collapsed and the plasmon resonance band characteristic of monodispersed nanoparticles appeared at ∼420 nm. Color changes in the colloidal solution were monitored by visual inspection. Digital images of the samples were captured with a digital still camera (Cannon-550D) at an optical zoom of 4×. The presence of Ce in the Ce-Ce-nGel was investigated using EDX. The morphology of Ce-nGel particles was observed under a TECNAI TEM (Fei, Electron Optics) HRTEM operated at 200 kV equipped with Olympus Soft Imaging Solutions GmbH (software: iTEM; TEM Camera: Morada 4008 × 2672 pixel max) recording system. For HRTEM analysis, the samples were prepared by placing one drop of the aqueous nGel on a carbon-coated copper TEM grid and dried at room temperature. The average diameter and size distribution were calculated from 50 readings of the images. Dynamic light scattering based on the concept of laser light scattering by particles in constant Brownian motion was employed to analyze the particle size. A high-performance DLS instrument (Beckmann Coulter DelsaTM Nano) was used for the size determination of Ce-nGel in the wet stage. The average values of the particle size and polydispersity, defined as a relative width of the size distribution, were determined from the DLS measurements.

The article "Cerium oxide nanoparticle-loaded polyvinyl alcohol nanogels delivery for wound healing care systems on surgery" was retracted in 2023. Reasons: lack of ethics approval or compliance; concerns about the data; concerns about the results or conclusions.

### 2.4. Synthesis of Ce-nGel and Ce-nGel-Glu nanocomposites for bandaging

A dip-coating technique was employed to fabricate Ce-nGel and Ce-nGel-Glu composite dressings. Briefly, the cotton fabric was dipped into the Ce-nGel and Ce-nGel-Glu nanogel, taken out, and dried at 50 °C for 24 h. The moisture content of nGel coated fabrics was measured as follows. A 3 × 3 cm^2^ sample of Ce-nGel coated fabric was weighed accurately and then dried at 105 °C for 4 h. The dried fabric sample was conditioned at 65% relative humidity in a desiccator for 24 h and reweighed.

### 2.5. Detection of Ce contents

The Ce content in Ce-nGel coated cotton fabrics was measured according to the previous method. Dried coated fabric of size (2 × 2) unit in cm^2^ was immersed in 30 mL of 15% nitric acid for 2 h. Cerium concentration was recorded by using Perkin Elmer Lambda 3100 flame atomic absorption spectrometer (AAS) equipped with a silver lamp at 328 nm.

### 2.6. Controlled release profile of Ce

In vitro Cerium release studies were performed at 37 °C using a Franz diffusion cell with separate donor and receptor compartments. The receptor compartment, which has a capacity of 30 mL, was filled with phosphate-buffered saline solution (pH 7.4). Nylon net was mounted between the donor and receptor compartments. Ce-nGel loaded fabric sample of 2 × 2 cm^2^ size was placed over the nylon net so that it is in contact with the medium of the receptor compartment at all times. The Cerium release pattern was obtained by sampling 3 mL aliquots from the receptor compartment solution at predetermined time intervals over a period of 48 h. The receptor compartment was replenished with an equal volume of phosphate buffer every time a sample was withdrawn. Each experiment was repeated three times. AAS analysis was carried out to detect the Cerium content in each aliquot. The cumulative amount of Cerium permeated per square centimeter of fabric sample was plotted against time. (Kim & Lee, 2017; Montaser et al., 2019; Shefa et al., 2020).

The article "Cerium oxide nanoparticle-loaded polyvinyl alcohol nanogels delivery for wound healing care systems on surgery" was retracted in 2023. Reasons: lack of ethics approval or compliance; concerns about the data; concerns about the results or conclusions.

### 2.7. Antibacterial properties of Ce-nGel and Ce-nGel-Glu

Antibacterial studies of dressings were carried out by colony count and zone inhibition methods, according to test method AATCC 100–1998. The antibacterial efficiency of Ce-nGel and Ce-nGel-Glu dressings was monitored against Gram positive bacteria *S. aureus* and Gram negative bacteria *E. coli*. The nanogel samples were added to the culture dishes and maintained at 37 °C for 24 h. The marked phases of the flexible microbes were quantified in the same manner as the microbes with the saline and agar plates. Bacterial growth rates were examined using statistical models.

### 2.8. Cell viability of Ce-nGel and Ce-nGel-Glu

The cell viability in the synthesized hydrogel was evaluated using the NIH-3T3 fibroblasts by Alamar Blue assay. The sterilized samples were placed in 96-well plates with the same fluency as the fibroblasts. The cells were marked for three different days. Cell viability was measured at 520 nm using a microplate reader. The experiments were repeated three times.

### 2.9. Animal experiments of the wound bandaging model

Male Swiss albino mice of Balb/C strain weighing 25–30 g were used for the wound healing experiments. Animals were acclimatized for 7 days prior to the start of experiments in the laboratory housing conditions of 26 ± 2 °C, 60–70% RH and 12 h light and dark cycle. All the experimental procedures and protocols used in this study were approved by the Institutional Animal Ethical Committee (Animal models), Emergency Department, Dongying People's Hospital, Dongying 257091, Shandong, China. The wounds were covered with the baseline damage and used as the negative control (Group I), nanogel-loaded bandaging (Group II), Ce-nGel (Group III), and Ce-nGel-Glu (Group IV). The extent of wound closure was analyzed by drawing the wound boundary at the end of 0, 4, 8, 16, and 24 days. The wounds closure was expressed in mm^2^. The wounds area was calculated using previously reported methods.

### 2.10. Statistical analysis

All inventory data are uttered as the mean ± standard deviations. Significant changes among groups were examined using one-way examination of modification, and changes for separate groups were dogged using Student’s *t* tests. The outcomes were observed as a significant difference when *p* < .05.

## 3. Results and discussion

### 3.1. Fabrication and characterization

By employing an easy and effective method to fabricate CeNPs, the current study aimed at using PVA as a stabilizing agent as well as a hydrogel system for the encapsulation of CeNPs. To avoid the clusters collisions and their growing into macro nanoparticles, the hydroxy fragments of PVA interact with the CeNPs and aid in steadying them and preventing their agglomeration and further proliferation. The graphical representation of the generation and anchoring of CeNPs within a PVA nanogel matrix is depicted in Figure 1.

The article "Cerium oxide nanoparticle-loaded polyvinyl alcohol nanogels delivery for wound healing care systems on surgery" was retracted in 2023. Reasons: lack of ethics approval or compliance; concerns about the data; concerns about the results or conclusions.

**Figure 1.** Schematic representation of Ce-nGel and Ce-nGel-Glu synthesis and its applications.

The morphology was observed by SEM and HR-TEM. (Figure 2(A,C)). The EDX spectra show distinctive energy peaks at ∼0.2 keV and SPR of C and O with stable peaks at ∼3 keV, indicating the presence of Ce. The contents of C, O, and Ce were measured to be 20.2%, 42.5%, and 38.1%, correspondingly. The formation of Ce-nGel was found to be markedly precious by the situations of the reduction reaction (Figure 2(B)). The TEM images show spherically shaped CeNPs. The TEM images correspond to the DLS analysis results (Figure 2(C)). The Cerium contents in the Ce-nGel were investigated by EDX analysis, as shown in Figure 2(B). The time-dependent difference in DLS analysis shows the particle size and diameters of the nanoparticles (Figure 2(E)). The role of PVA is to stabilize the nanoparticle formation and provide the base matrix for the nanogels. It was observed that the average particle size of the Ce-nGel was in the range of 90–150 nm for a reaction duration of up to 20 min.

**Figure 2.** Preparation and characterization of Ce-nGel and Ce-nGel-Glu nanocomposites for bandaging. (A) SEM image of Ce-nGel. (B) EDX studies of Ce-nGel. (C) TEM images of nGel with reaction time of 120 min. Scale bar, 200 nm. (D) UV-visible studies of Ce-nGel with reaction time 5 min (black), 20 min (blue), 60 min (orange), and 120 min (pink). (E) Variation in particle size of Ce-nGel with the reaction time. (F) Cerium release study of Ce-nGel with time. Conditions: Cerium content, 5.75 µg/cm^2^; release temperature, 37 °C; pH, 7.2.

The UV-Vis spectrum confirmed the presence of CeNPs (Figure 2(D)). Normally, CeNPs exhibit versatile and changeable optical property that depends on their size and shape. The formation of CeNPs was examined at different time intervals with the SPR band observed between 400 and 450 nm at 5 min of reduction time. From 10 min to 120 min, the intensity of the peak increased with slight changes in the maximum absorption, owing to the variations in the size of the nanoparticles. After 120 min, there was no noticeable difference in the plasma intensity band of the CeNPs perceived at 420 nm, suggesting the achievement of the decrease reaction at 120 min.

The article "Cerium oxide nanoparticle-loaded polyvinyl alcohol nanogels delivery for wound healing care systems on surgery" was retracted in 2023. Reasons: lack of ethics approval or compliance; concerns about the data; concerns about the results or conclusions.

### 3.2. Fabrication of Ce-nGel and Ce-nGel-Glu nanocomposites for bandaging

Cotton fabric was used as the permeable support substrate to attach Ce-nGel and Ce-nGel-Glu. It has wide acceptability over other textiles due to its natural abundance and intrinsic properties, such as hydrophilicity, better conduction of heat, and comfortable feel. Therefore, commercial cotton fabric was chosen in this work for the coating process. The fabric samples were dipped into the Ce-nGel and Ce-nGel-Glu solutions and dried at 50 °C. The interaction between the fabric and the colloidal solution coating results from the physical adsorption of nanogels on the fabric surface. The add-on on cotton varied in the range of 0.8–3.2% as the number of dip coatings increased from one to four. It was observed that the dressings exhibited slightly enhanced rigidity as the add-on content increased.

### 3.3. Controlled release profile of Cerium

From the surface plasmon band results, it was inferred that the chemical reduction process at 80 °C and a reaction time of 60 min leads to the formation of nanogels with the least and regular size. As a result, this sample was chosen to analyze the cumulative Cerium release from the Ce-nGel coated dressing. The amount of Cerium theoretically available for release and the actual amount of Cerium (free ionic Cerium or the neutral Cerium nanoparticles) were measured after digestion of the Ce-nGel dressing in HNO_3_. The cumulative release of Cerium from Ce-nGel coated dressing after immersion in PBS solution was also determined. As shown in Figure 2(F), the release of Cerium is rapid in the beginning, and then it becomes slower after 16 h. The Cerium release continued further to 48 h at a slow rate. The Cerium content in the sample was found to be 5.48 µg/cm^2^. However less than half of the actual amount (∼2 µg/cm^2^) of Cerium leached out from the dressing after 48 h. The slow release is the indication of atomic Cerium leaching out as Cerium ions in the medium.

### 3.4. Ce-nGel-Glu surface morphology

Surface morphology and topography of the dressings at different stages was studied by SEM and AFM, respectively. SEM analysis results are presented in Figure 3. Figure 3 show SEM images of the uncoated fabric at different magnifications and the surface appears to be smooth. Figure 3 shows SEM images of the Ce-nGel dressing. The higher magnification images indicate the presence of homogeneous coating of the nanogel and also the deposition of nanoparticles on the dressing surface. Figure 3 reveals the surface morphology of Ce-nGel-Glu dressing. The addition of glycerol to Ce-nGel induces a drastic change in the surface morphology of the coated fabric with some convoluted shell-like structures on the surface. Glycerol increases the flexibility and moisturized nature of the dressing while the sticky nature would facilitate easy removal from the wound site. After Cerium release, the morphologies were observed to be vastly different than prior to release as shown in Figure 3. The SEM images show a massive presence of Cerium oxide crystals on the dressing. After Cerium release the dressing surface becomes rough due to leaching of the components (Cerium and glycerol) and salt deposition.

The article "Cerium oxide nanoparticle-loaded polyvinyl alcohol nanogels delivery for wound healing care systems on surgery" was retracted in 2023. Reasons: lack of ethics approval or compliance; concerns about the data; concerns about the results or conclusions.

**Figure 3.** SEM images of pure fabric, Ce-nGel, Ce-nGel-Glu, and Ce-nGel dressings after washing. Scale bar: pure fabric (40 µM), Ce-nGel (10 µM), Ce-nGel-Glu (10 µM), and Ce-nGel dressings after washing (10 µM).

### 3.3. Mechanical properties

To confirm the integrity of the membranes, the mechanical properties of the hydrogel and nanocomposite are important for effective dressing applications. The mechanical properties (tensile strength, maximum elongation, and tensile modulus) of the pure materials (Ce-nGel-Glu), the as-prepared Ce-nGel and Ce-nGel-Glu are illustrated in Figure 4(A). It is noted that the addition of CeNPs to the Ce-nGel-Glu had a variable effect on the tensile strength and total elongation. The Ce-nGel and Ce-nGel-Glu exhibited a tensile strength of 2.2 ± 0.6 and 2.9 ± 0.4 MPa, respectively, which was sufficient for tissue covering the wound. (Figure 4(B)). The improved tensile strength ensures greater fracture toughness of the samples. These results demonstrated that the Ce-nGel nanocomposite have good mechanical properties suitable for use in biomedical applications. The elongation at break values represent the flexibility of the nGel and Ce-nGel bandage. Pure CeNPs, Ce-nGel and Ce-nGel-Glu, the as-prepared Ce-nGel exhibited an elongation in the range from 20% to 50% at the fracture points (Figure 4(C)). Figure 4 also shows that the tensile strength increased with an increase in Ce concentration. The result of the tensile modulus (Figure 4(D)) was consistent with the stress test. Overall, Ce-nGel demonstrated higher tensile modulus and elongation than CeNPs, Ce-nGel and Ce-nGel-Glu, however it exhibited lower maximum strength. Therefore, flexibility would be an important consideration for the application of Ce-nGel-Glu nanocomposites for various types of wound surface.

**Figure 4.** Mechanical properties comparison of (A) Stress-strain curve. (B) Tensile strength. (C) Elongation. (D) Tensile modulus of CeNPs, Ce-nGel and Ce-nGel-Glu nanocomposite.

### 3.4. Biodegradation and swelling studies

Hydrogels have become the subject of improvement for use in many applications. The percentage weight loss (Figure 5(A)) revealed limited degradation of the Ce-nGel-Glu bandages. All the as-fabricated bandages showed a degradation of 24–27% (1 day), 39–48% (4 days) and 75–84% (7 days) after immersion in PBS medium, respectively. The presence of CeNPs reduced the degradation rate in the composite bands. This can be attributed to the interaction between the CeNPs, Ce-nGel and Ce-nGel-Glu bandages. However, the as-fabricated bandage was degraded in vitro, while retaining its characteristics and form even after the 7th day in a situation without agitation of degradation behavior. The swelling of the Ce-nGel and Ce-nGel-Glu dressings were examined after 1, 4 and 7 days of incubation in PBS medium (Figure 5(B)). Figure 5(B) suggested that Ce-nGel-Glu exhibited higher swelling capacity compared to pure Ce-nGel hydrogel bandages. Furthermore, the nGel and Ce-nGel-Glu bandages showed similar swelling activity even after the addition of CeNPs. An improvement in the swelling ability of Ce-nGel-Glu can be attributed to the presence of CeNPs nanoparticles of different sizes, morphology and surface charges. Additionally, the formation of CeNPs nanoparticles can cause the Ce-nGel-Glu to expand, thereby expanding the pores and free spaces in the Ce-nGel-Glu, which would thereby absorb more water.

The article "Cerium oxide nanoparticle-loaded polyvinyl alcohol nanogels delivery for wound healing care systems on surgery" was retracted in 2023. Reasons: lack of ethics approval or compliance; concerns about the data; concerns about the results or conclusions.

**Figure 5.** (A) Biodegradation and (B) Swelling ratio as-fabricated bandages of CeNPs, Ce-Ce-nGel and Ce-nGel-Glu nanocomposite using different days (1, 4, and 7) of activity.

### 3.5. Antibacterial and cell viability analyses

The antibacterial properties of the fabricated Ce-nGel and Ce-nGel-Glu dressings were investigated using *S. aureus* (gram-positive microbe) and *E. coli* (gram-negative microbe), and the results are shown in Figure 6(A). In our previous studies, the Ce-nGel-Glu dressings exhibited higher antibacterial activity with both microbes compared to Ce-nGel. The bacterial property of Ce-nGel-Glu was reduced by the presence of free Ce-nGel (Ali & Ahmed, 2018; Hsu et al., 2020; Kuddushi et al., 2020).

**Figure 6.** Antibacterial and cell viability examinations. (A) Colony formation of *S. aureus* and *E. coli*. (B) Cell viability of Ce-nGel and Ce-nGel-Glu. The experiments were repeated three times. Scale bar 40 µm. Values are expressed as the mean ± SD. *p < .05, **p < .01.

The outcomes of cell viability established that Cerium (positive control) and Ce-nGel (control) did not demonstrate any harm on days 1, 3, and 7 in development with NIH-3T3 fibroblasts (Figure 6(B)). The synthesized Ce-nGel-Glu dressings showed ∼75% viability after day 1 of culture, which further increased up to ∼93% after 3 and 7 days of development. The reduced cell viability on day 1 was due to the presence of free Ce-nGel with the NIH3T3 fibroblasts. After day 1, the remaining viable fibroblasts multiplied, consequently improving the viability (Subarkhan & Ramesh, 2016; Mohamed Kasim et al., 2018; Mohamed Subarkhan et al., 2019; Balaji et al., 2020; Sathiya Kamatchi et al., 2020).

The article "Cerium oxide nanoparticle-loaded polyvinyl alcohol nanogels delivery for wound healing care systems on surgery" was retracted in 2023. Reasons: lack of ethics approval or compliance; concerns about the data; concerns about the results or conclusions.

### 3.6. *In vivo* examination of CeNPs

The procedure for the application of dressing on the mouse wound is depicted in Figure 7. The dressing beyond the wound area was fixed by using an adhesive tape so that the dressing stays in contact with the wound. The wound healing performance of various samples on Swiss albino mice is presented in Figure 7, at different time intervals (0, 6, 12, and 24). The reduction in wound area was calculated. The wound treatment with control fabric showed only 50% wound reduction after 12 days while gel-coated dressing showed 70% wound healing. nGel treated wounds were much smaller, with 80% wound closure being achieved in 24 days. In the case of Ce-nGel-Glu treated mice, almost complete healing was observed in 24 days. This enhanced rate of wound healing is attributed to the faster leaching of Cerium from the dressing due to the presence of glycerol. The Cerium nanoparticles which are released from the matrix slowly change to Ce^+^ under physiological conditions and interact with bacterial cells present at the wound site. The Ce^+^ concentration obtained from the sustained release is well within the safety limits and thus, damage to normal human cells is avoided. Winter reported that epithelialization is retarded by the dry scab and that epithelialization can be accelerated if the wound is kept moist. One explanation for this was that keratinocytes migrated more easily over a moist wound surface than underneath a scab. This is the reason why wound reduction of the Ce-nGel-Glu treated wound was higher than that of without glycerol on the 24th day. No scab and argyria were observed for the wounds treated with nGel and Ce-nGel-Glu dressings. In the case of control, gauze adhered to the wound, causing damage each time it was replaced. By gross examination of the wound sites, it may also be inferred that scar formation is minimum when wounds were treated with Ce-nGel and Ce-nGel-Glu composite dressings (Das & Subuddhi, 2013; Singh & Dhiman, 2015; Yadav et al., 2019).

**Figure 7.** Photographs of an *in vivo* wound healing study. (A) Extent of closure of wounds treated with control, Ce-nGel, and Ce-nGel-Glu. (B) Evaluation of the wound area shutter. The values are expressed as the mean ± SD. *p < .05, **p < .01.

The article "Cerium oxide nanoparticle-loaded polyvinyl alcohol nanogels delivery for wound healing care systems on surgery" was retracted in 2023. Reasons: lack of ethics approval or compliance; concerns about the data; concerns about the results or conclusions.

### 3.7. Histological evaluation

Histological analysis is a powerful method to observe the progress in healing and tissue regeneration of wounds (Sonamuthu et al., 2020). Histological analysis focused on the healing ability of injured mice tissues due to the influence of hematoxylin and eosin (H&E) staining on the Ce-nGel (control) and Ce-nGel-Glu (Figure 8). The Ce-nGel-Glu showed excellent healing after day 0, 6, 12 and 24, in contrast to the bare wound. In Figure 8, the histological sections indicated compact keratinocytes in the epidermis on wounds coated with Ce-nGel and Ce-nGel-Glu, compared to the bare wound. In addition, the existence of Ce-nGel-Glu also improved the healing rate of Ce-nGel coated wounds, which was evident from the histological micrographs. The biocompatibility and anticoagulant properties of CeNPs nanoparticles make it an excellent candidate for wound healing, as seen in *in vitro* and *in vivo* studies. Conversely, absolute regrowth of new subcutaneous tissues was quantitated by segment light microscopy. The degree of wound closure was estimated macroscopically. After 6 and 12 days, wounds dressed in the Ce-nGel and Ce-nGel-Glu achieved a large closure of around 95%, in contrast to 65% wound closure of the bare wounds (Figure 8). Therefore, *in vivo* study of Sprague-Dawley rats confirmed the increased wound healing ability of the as-fabricated Ce-nGel-Glu (Ghobril & Grinstaff, 2015; Sethuram et al., 2019; Zhang et al., 2020).

**Figure 8.** (A) Photomicrographs H&E-stained control, as-fabricated bandages of control, Ce-Ce-nGel and Ce-nGel-Glu hydrogel nanocomposite treated wounds. Scale bar 20 µm.

## 4. Conclusion

Our study aimed at developing novel wound bandages by covering nanogels loaded with CeNPs on the surface of cotton fabrics. Herein, cotton acts as a supporting layer for the nanogel. Well-dispersed CeNPs are generated with the stabilizing effect of PVA as the nanogel medium. The nanogel thus formed had a size in the series of ∼10–50 nm. Together Ce-nGel and Ce-nGel-Glu nanocomposite bandages showed significant antibacterials properties even at low absorptions. A slow rate of releases was detected for the nanogels bandages with ∼2 µg/cm^2^ of Ce leaking out in 48 h. These low attentions of Ce are very nontoxic for the human body. The Ce-nGel-Glu bandaging displayed 100% closure of full width wound by day 24, which may be because the occurrence of glycerol quickens the release of Ce from the medium, therefore assisting wounds closure. The wound bandages might be effortlessly exposed off from the wounds sites without affecting the tissues. The results of these investigations suggest that Ce-nGel-Glu could be a promising wounds care composition having effective damage and scar prevention.

The article "Cerium oxide nanoparticle-loaded polyvinyl alcohol nanogels delivery for wound healing care systems on surgery" was retracted in 2023. Reasons: lack of ethics approval or compliance; concerns about the data; concerns about the results or conclusions.

## References

[CIT0001] Ali A, Ahmed S. (2018). Recent advances in edible polymer based hydrogels as a sustainable alternative to conventional polymers. J Agric Food Chem 66:6940–67.2987876510.1021/acs.jafc.8b01052

[CIT0002] Bakshi MS. (2017). Nanotoxicity in systemic circulation and wound healing. Chem Res Toxicol 30:1253–74.2847867710.1021/acs.chemrestox.7b00068

[CIT0003] Balaji S, Mohamed Subarkhan MK, Ramesh R, et al. (2020). Synthesis and structure of arene Ru(II) N∧O-chelating complexes: *in vitro* cytotoxicity and cancer cell death mechanism. Organometallics 39:1366–75.

[CIT0004] Das S, Subuddhi U. (2013). Cyclodextrin mediated controlled release of naproxen from pH-sensitive chitosan/poly(vinyl alcohol) hydrogels for colon targeted delivery. Ind Eng Chem Res 52:14192–200.

[CIT0005] Deal HE, Brown AC, Daniele MA. (2020). Microphysiological systems for the modeling of wound healing and evaluation of pro-healing therapies. J Mater Chem B 8:7062–75.3275671810.1039/d0tb00544dPMC7460719

[CIT0006] Deng Z, Wang H, Ma PX, et al. (2020). Self-healing conductive hydrogels: preparation, properties and applications. Nanoscale. Royal Soc Chem 12:1224–46.10.1039/c9nr09283h31859313

[CIT0007] Gao Y, Li Z, Huang J, et al. (2020). In situ formation of injectable hydrogels for chronic wound healing. J Mater Chem B 8:8768–80.3302638710.1039/d0tb01074j

[CIT0008] Ghobril C, Grinstaff MW. (2015). The chemistry and engineering of polymeric hydrogel adhesives for wound closure: a tutorial. Chem Soc Rev 44:1820–35.2564926010.1039/c4cs00332b

[CIT0009] Hamdan S, Pastar I, Drakulich S, et al. (2017). Nanotechnology-driven therapeutic interventions in wound healing: potential uses and applications. ACS Cent Sci 3:163–75.2838659410.1021/acscentsci.6b00371PMC5364456

[CIT0010] Hartwell R, Leung V, Chavez-Munoz C, et al. (2011). A novel hydrogel-collagen composite improves functionality of an injectable extracellular matrix. Acta Biomater 7:3060–9.2156987010.1016/j.actbio.2011.04.024

[CIT0011] Hsu HH, Liu Y, Wang Y, et al. (2020). Mussel-inspired autonomously self-healable all-in-one supercapacitor with biocompatible hydrogel. ACS Sustainable Chem Eng 8:6935–48.

[CIT0012] Hu H, Xu F-J. (2020). Rational design and latest advances of polysaccharide-based hydrogels for wound healing. Biomater Sci 8:2084–101.3211824110.1039/d0bm00055h

[CIT0013] Kim J, Lee C-M. (2017). Wound healing potential of a polyvinyl alcohol-blended pectin hydrogel containing Hippophae rahmnoides L. extract in a rat model. Int J Biol Macromol 99:586–93.2828345110.1016/j.ijbiomac.2017.03.014

[CIT0014] Kuddushi M, Ray D, Aswal V, et al. (2020). Poly(vinyl alcohol) and functionalized ionic liquid-based smart hydrogels for doxorubicin release. ACS Appl Bio Mater 3:4883–94.10.1021/acsabm.0c0039335021732

The article "Cerium oxide nanoparticle-loaded polyvinyl alcohol nanogels delivery for wound healing care systems on surgery" was retracted in 2023. Reasons: lack of ethics approval or compliance; concerns about the data; concerns about the results or conclusions.

[CIT0015] Liang Y, Zhao X, Hu T, et al. (2019). Adhesive hemostatic conducting injectable composite hydrogels with sustained drug release and photothermal antibacterial activity to promote full-thickness skin regeneration during wound healing. Small 15:1900046.10.1002/smll.20190004630786150

[CIT0016] Liang Y, Chen B, Li M, et al. (2020). Injectable antimicrobial conductive hydrogels for wound disinfection and infectious wound healing. Biomacromolecules 21:1841–52.3238899810.1021/acs.biomac.9b01732

[CIT0017] Liu H, Wang C, Li C, et al. (2018). A functional chitosan-based hydrogel as a wound dressing and drug delivery system in the treatment of wound healing. RSC Adv 8:7533–49.3553913210.1039/c7ra13510fPMC9078458

[CIT0018] Ma Z, Song W, He Y, et al. (2020). Multilayer injectable hydrogel system sequentially delivers bioactive substances for each wound healing stage. ACS Appl Mater Interfaces 12:29787–806.3251557710.1021/acsami.0c06360

[CIT0019] Memic A, Abudula T, Mohammed HS, et al. (2019). Latest progress in electrospun nanofibers for wound healing applications. ACS Appl Bio Mater 2:952–69.10.1021/acsabm.8b0063735021385

[CIT0020] Mohamed Kasim MS, Sundar S, Rengan R. (2018). Synthesis and structure of new binuclear ruthenium(II) arene benzil bis(benzoylhydrazone) complexes: investigation on antiproliferative activity and apoptosis induction. Inorg Chem Front 5:585–96.

[CIT0021] Mohamed Subarkhan MK, Ren L, Xie B, et al. (2019). Novel tetranuclear ruthenium(II) arene complexes showing potent cytotoxic and antimetastatic activity as well as low toxicity *in vivo*. Eur J Med Chem 179:246–56.3125592510.1016/j.ejmech.2019.06.061

[CIT0022] Montaser AS, Rehan M, El-Naggar ME. (2019). pH-Thermosensitive hydrogel based on polyvinyl alcohol/sodium alginate/N-isopropyl acrylamide composite for treating re-infected wounds. Int J Biol Macromol 124:1016–24.3050049410.1016/j.ijbiomac.2018.11.252

[CIT0023] Nethi SK, Das S, Patra CR, et al. (2019). Recent advances in inorganic nanomaterials for wound-healing applications. Biomater Sci 7:2652–74.3109437410.1039/c9bm00423h

[CIT0024] Qu J, Zhao X, Liang Y, et al. (2018). Antibacterial adhesive injectable hydrogels with rapid self-healing, extensibility and compressibility as wound dressing for joints skin wound healing. Biomaterials 183:185–99.3017224410.1016/j.biomaterials.2018.08.044

[CIT0025] Sakai S, Tsumura M, Inoue M, et al. (2013). Polyvinyl alcohol-based hydrogel dressing gellable on-wound via a co-enzymatic reaction triggered by glucose in the wound exudate. J Mater Chem B 1:5067–75.3226109710.1039/c3tb20780c

The article "Cerium oxide nanoparticle-loaded polyvinyl alcohol nanogels delivery for wound healing care systems on surgery" was retracted in 2023. Reasons: lack of ethics approval or compliance; concerns about the data; concerns about the results or conclusions.

[CIT0026] Sathiya Kamatchi T, Mohamed Subarkhan MK, Ramesh R, et al. (2020). Investigation into antiproliferative activity and apoptosis mechanism of new arene Ru(ii) carbazole-based hydrazone complexes. Dalton Trans 49:11385–95.3277604210.1039/d0dt01476a

[CIT0027] Sekhon UDS, Sen Gupta A. (2018). Platelets and platelet-inspired biomaterials technologies in wound healing applications. ACS Biomater Sci Eng 4:1176–92.3341865510.1021/acsbiomaterials.7b00013

[CIT0028] Sener G, Hilton SA, Osmond MJ, et al. (2020). Injectable, self-healable zwitterionic cryogels with sustained microRNA – cerium oxide nanoparticle release promote accelerated wound healing. Acta Biomater 101:262–72.3172625010.1016/j.actbio.2019.11.014

[CIT0029] Sethuram L, Thomas J, Mukherjee A, et al. (2019). Effects and formulation of silver nanoscaffolds on cytotoxicity dependent ion release kinetics towards enhanced excision wound healing patterns in Wistar albino rats. RSC Adv 9:35677–94.3552807010.1039/c9ra06913ePMC9074428

[CIT0030] Shefa AA, et al. (2020). Curcumin incorporation into an oxidized cellulose nanofiber-polyvinyl alcohol hydrogel system promotes wound healing. Mate Des 186:108313.

[CIT0031] Shen T, Dai K, Yu Y, et al. (2020). Sulfated chitosan rescues dysfunctional macrophages and accelerates wound healing in diabetic mice. Acta Biomater 117:192–203.3300748610.1016/j.actbio.2020.09.035

[CIT0032] Singh B, Dhiman A. (2015). Designing bio-mimetic moxifloxacin loaded hydrogel wound dressing to improve antioxidant and pharmacology properties. RSC Adv 5:44666–78.

[CIT0033] Son YJ, Tse JW, Zhou Y, et al. (2019). Biomaterials and controlled release strategy for epithelial wound healing. Biomater Sci 7:4444–71.3143626110.1039/c9bm00456d

[CIT0034] Sonamuthu J, Cai Y, Liu H, et al. (2020). MMP-9 responsive dipeptide-tempted natural protein hydrogel-based wound dressings for accelerated healing action of infected diabetic wound. Int J Biol Macromol 153:1058–69.3175648610.1016/j.ijbiomac.2019.10.236

[CIT0035] Song DW, Kim SH, Kim HH, et al. (2016). Multi-biofunction of antimicrobial peptide-immobilized silk fibroin nanofiber membrane: implications for wound healing. Acta Biomater 39:146–55.2716340410.1016/j.actbio.2016.05.008

[CIT0036] Subarkhan MKM, Ramesh R. (2016). Ruthenium(ii) arene complexes containing benzhydrazone ligands: synthesis, structure and antiproliferative activity. Inorg Chem Front 3:1245–55.

[CIT0037] Thakar H, Sebastian SM, Mandal S, et al. (2019). Biomolecule-conjugated macroporous hydrogels for biomedical applications. ACS Biomater Sci Eng 5:6320–41.3341780810.1021/acsbiomaterials.9b00778

The article "Cerium oxide nanoparticle-loaded polyvinyl alcohol nanogels delivery for wound healing care systems on surgery" was retracted in 2023. Reasons: lack of ethics approval or compliance; concerns about the data; concerns about the results or conclusions.

[CIT0038] Thapa RK, Diep DB, Tønnesen HH. (2020). Topical antimicrobial peptide formulations for wound healing: current developments and future prospects. Acta Biomater 103:52–67.3187422410.1016/j.actbio.2019.12.025

[CIT0039] Thongsuksaengcharoen S, Samosorn S, Songsrirote K. (2020). A facile synthesis of self-catalytic hydrogel films and their application as a wound dressing material coupled with natural active compounds. ACS Omega 5:25973–83.3307312410.1021/acsomega.0c03414PMC7558030

[CIT0040] Tu Y, Chen N, Li C, et al. (2019). Advances in injectable self-healing biomedical hydrogels. Acta Biomater 90:1–20.3095189910.1016/j.actbio.2019.03.057

[CIT0041] Wang K, Nune KC, Misra RDK. (2016). The functional response of alginate-gelatin-nanocrystalline cellulose injectable hydrogels toward delivery of cells and bioactive molecules. Acta Biomater 36:143–51.2697166510.1016/j.actbio.2016.03.016

[CIT0042] Xu C, Dai G, Hong Y. (2019). Recent advances in high-strength and elastic hydrogels for 3D printing in biomedical applications. Acta Biomater 95:50–9.3112572810.1016/j.actbio.2019.05.032PMC6710142

[CIT0043] Yadav TC, Srivastava AK, Mishra P., et al. (2019). ‘Electrospinning: an efficient biopolymer-based micro- and nanofibers fabrication technique’, in *Next Generation Biomanufacturing Technologies*. Am Chem Soc 10:209.

[CIT0044] Yu H, Peng J, Xu Y, et al. (2016). Bioglass activated skin tissue engineering constructs for wound healing. ACS Appl Mater Interfaces. 8:703–15.2668471910.1021/acsami.5b09853

[CIT0045] Zhang C, Wu B, Zhou Y, et al. (2020). Mussel-inspired hydrogels: from design principles to promising applications. Chem Soc Rev 49:3605–37.3239393010.1039/c9cs00849g

[CIT0046] Zhao X, Liu L, An T, et al. (2020a). A hydrogen sulfide-releasing alginate dressing for effective wound healing. Acta Biomater 104:85–94.3190145610.1016/j.actbio.2019.12.032

[CIT0047] Zhao X, Liang Y, Huang Y, et al. (2020b). Physical double-network hydrogel adhesives with rapid shape adaptability, fast self-healing, antioxidant and NIR/pH stimulus-responsiveness for multidrug-resistant bacterial infection and removable wound dressing. Adv Funct Mater 30:1910748.

